The article "A Simple-to-Use Nomogram for Predicting Survival in Children with Acute Myeloid Leukemia" was published in 2021. Journal: Biomed Res Int.

# A Simple-to-Use Nomogram for Predicting Survival in Children with Acute Myeloid Leukemia

**DOI:** 10.1155/2021/7264623

**Published:** 2021-03-11

**Authors:** Feng Jiang, Xiang Yu, Chuyan Wu, Ming Wang, Ke Wei, Guoping Zhou, Jimei Wang

**Affiliations:** ^1^Department of Pediatrics, The First Affiliated Hospital of Nanjing Medical University, Nanjing 210029, China; ^2^Neonatal Department, Obstetrics and Gynecology Hospital of Fudan University, Shanghai 200011, China; ^3^Department of Rehabilitation Medicine, The First Affiliated Hospital of Nanjing Medical University, Nanjing 210029, China; ^4^Department of Plastic and Burn Surgery, The First Affiliated Hospital of Nanjing Medical University, Nanjing 210029, China; ^5^Medical Service Section, The First Affiliated Hospital of Nanjing Medical University, Nanjing 210029, China

## Abstract

**Background:**

The research analyzed a group of patients to develop a statistical nomogram and a web-based survival rate predictor for the comprehensive estimate of the overall survival (OS) of children with acute myeloid leukemia.

**Methods:**

Between 1999 to 2015, we used the Therapeutically Applicable Research to Generate Effective Treatments (TARGET) database to evaluate and randomly divide 440 children diagnosed with AML into the population of training (*n* = 309) and validation (*n* = 131). The analysis of Lasso Cox was used to identify separate predictive variables. We have used essential forecasting considerations to construct a nomogram and a web-based calculator focused on Cox regression analysis. Nomogram validation was tested through discrimination and calibration.

**Results:**

Compared to the multivariate training cohort models, a nomogram integrating gender, age of diagnose, WBC at diagnosis, bone marrow leukemic blast percentage, and chromosomal abnormalities [*t*(8; 21), inv(16)] were designed for the prediction of OS. We also developed a predictive survival nomogram and a web-based calculator. C-indexes validated internally and checked externally were 0.747 and 0.716. The calibration curves have shown that the nomogram might accurately forecast 3-year and 5-year OS.

**Conclusions:**

A nomogram effectively predicts survival in children with AML. This prognostic model can be used in clinical practice.

## 1. Background

Acute myeloid leukemia (AML) is a disease of the hematopoietic stem cells (HSC), marked by irregular development and immature blast cell proliferation in the bone marrow [1, 2]. Childhood AMLs account for nearly 20% of childhood leukemia and >50% of fatalities in the aforementioned populations [3, 4]. Several contributing factors, including toxic exposures, chemotherapy or radiation treatment, myelodysplastic syndrome, and genetic factors, have led to AML pathogenesis [5–7]. Despite considerable progress in discovering pediatric AML pathophysiology, survival rates in patients have not significantly improved and nearly more than half of children diagnosed with AML suffering from recurrence.

In recent decades, AML has improved diagnosis and treatment but the overall survival rate (OS) is still low, less than 50% [8, 9]. The cytogenetic karyotype and molecular defects in the diagnosis are known to be the most important predictive factors for OS. Forecast probability stratification should be improved as it can establish successful diagnostic and therapeutic approaches.

Nomograms are accepted as a viable substitute method that can allow clinicians to accurately predict individuals [10, 11]. By adding clinically relevant variables, the survival rate can be measured accurately [12, 13]. Nevertheless, nomograms for the estimation of children's survival with AML have not yet been fully established.

In this research, we established a prognostic nomogram based on the TARGET population data to predict individualized survival in children with AML.

## 2. Methods

### 2.1. Patient Selection

We downloaded clinical information from the TARGET project database for AML patients (http://ocg.cancer.gov/). The criteria for AML were identified between 1999 and 2015. Criteria for exclusion were as follows: unclear gender, uncertain age of diagnose, unknown WBC at diagnosis, unknown bone marrow leukemic blast percentage (BM blast percentage), and unclear chromosomal results including *t*(8; 21), inv(16). As our mathematical research method, we used *R* software (3.5.2). The optimum diagnostic age cutoff value was 3489 days. 70% of all patients have been randomly chosen to form the Nomogram Construction Training Cohort, and the remaining 30% have been validated.

### 2.2. Ethical Approval

Because the identified patient information is not included in the TARGET database, no ethical consent is needed.

### 2.3. Training and Validation Cohort

The whole population was divided by the random sample process into the training or validation population (ratio, ~ 3 : 1). The training population was used to assess the predictive model and the statistical probability stratification. The validation population was used to verify the model prediction.

### 2.4. Statistical Analysis

Categorical measurements were represented as counts and percentages. Continuous measurements were represented as mean and range. The *t*-test was used to continuous measurements, while the Chi-square was used to compare ones. Statistically significant was *P* < 0.05. The primary endpoint was overall survival (OS). OS was described as an interval from diagnostic to death or last follow-up, regardless of the cause of death. The optimum age cutoff value was calculated by the *R* program package “survminer”.

We used the Lasso Cox regression model [14], defining individual operating system risk factors, as well as the “glmnet” package. Using the “rms package” program, nomograms and calibration plots were developed. We used the “shiny” and “DynNom” packages to create a web-based survival rate calculator that estimated overall survival rates (http://www.shinyapps.io/) dynamically. The nomogram measurement was carried out using the concordance index (C-index) and calibration curves. The C-index represents the nomogram's capacity to discriminate. The larger the C-index, the more accurate the model. For the analysis of the observed and predicted nomogram probabilities, calibration plots were used. The precision of the 3-year and 5-year nomogram survival was assessed by the ROC (receiver operating characteristic) curve.

## 3. Results

### 3.1. Patient Characteristics

In the TARGET database, we found 440 eligible patients (1999-2015). The median OS was 1547 days (range 1-3113 days). The OS rates for 3 years and 5 years were 70.9% and 44.3%, respectively. In Table 1, the demographic and clinical features of the population in training (*n* = 309), the validation population (*n* = 131), and all patients (*n* = 440) are illustrated.

### 3.2. Identification of Independent Risk Factors

Lasso Cox also used the training population to evaluate regression and classify individual risk factors impacting the OS (Figure 1). With increases in *λ,* the coefficient of variables decreased. The excluded variable parameters were compressed to 0 when *λ* was optimum. Variables < 0 have therefore been chosen. As a result, a total of 6 predictive factors (gender, age of diagnose, WBC at diagnosis, BM blast percentage, chromosomal abnormalities [*t*(8; 21), inv(16)]) were included in the predictive model. These factors were applied to the nomogram.

### 3.3. Nomogram

A nomogram that incorporates all the relevant independent factors was established for estimation of 3 years and 5 years OS, based on the reduced multivariate models of the training population (Figure 2). This model revealed the inv(16) translocation mainly contributed to the prognosis, followed by *t*(8; 21) translocation, WBC at diagnosis, age of diagnose, etc. Each factor received a score on the scale of points. By applying the scores to the overall scale, we might estimate the probability of 3-year and 5-year survival.

The calculator predicted patients' survival based on their clinical characteristics and based on these findings, we developed a dynamic web-based calculator (https://dxyjiang.shinyapps.io/AMLpredict/), to predict OS in AML patients by nomogram (Figure 3). For e.g., the OS rate for 5 years was approximately 96% for one patient aged 14, diagnosed with WBC of approximately 100 ≥ 10^9^/L, BM blast percentage ≥ 90%, and *t*(8; 21) and inv(16) positive.

### 3.4. Nomogram Validation

Internal analysis shows that the nomogram can estimate the OS correctly with a 0.747 C-index. Similarly, the external validation of the C-index was 0.716. The calibration statistics showed an outstanding correlation between the values for the 3-year and 5-year OS predicted and observed in both the population of training and the validation cohort (Figure 4).

### 3.5. Survival Curves for Prognostic Factors

Finally, we examined and developed curves of survival between the prognostic variables in the nomogram and the OS (Figure 5). We observed that age of diagnose, WBC at diagnosis, inv(16), and calculated risk scores wascorrelated with overall survival.

## 4. Discussion

As precision medicine develops quickly, physicians may create personalized diagnosis and follow-up plans for patients who need more accurate and easy models of survival [15, 16]. As a predictive tool, the nomogram can offer the most precise forecasts by means of a simple, easy to understand and easy to use in clinical procedure [17, 18]. The long-term survival of patients with various malignancies has been regularly estimated by demographic and clinical characteristics in a simple nomogram [19, 20].

AML is one of the most severe malignancies in childhood with different kinds of molecular and cellular heterogeneity [21, 22]. The standard cure of AML is the hematopoietic stem cell transplantation and chemotherapy, but the prognosis of childhood AML is suboptimal because of its elevated recurrence and mortality [23, 24]. Nomograms in recent research are typically more precise and convenient compared with conventional staging systems. In addition, web-based survival rate calculators were used to improve predictive model approachability. Recently, several reports have demonstrated nomograms for estimating AML adult patients' long-term survival outcomes [25, 26]. To our knowledge, few nomograms have been recorded to estimate the OS for children with AML. Hence, 440 patients were studied for the detection of OS-impact variables and a nomogram dependent calculator to effectively forecast prognostics for children with AML. Successful statistic evaluation was used to provide data for clinical consultation, pretreatment decision-making, and follow-up approaches.

The association between variables named multicollinearity has become a major issue in multivariate regression analysis [27]. We used the Lasso Cox regression approach rather than the conventional step-by-step process to tackle possible collinearity. The regression of Lasso Cox minimizes and reduces correlations thus offering a conclusive final model [28, 29].

The statistical model, which contained the aforementioned 13 individual risk factors, was extremely reliable in its survival prediction. C-index and validation plots have been used to test the predictive preciseness of the model and ensure the predictive precision of the nomogram. Both C-indices were >0.7 and demonstrated outstanding accuracy between predicted and actual survival. Nonetheless, given its high precision, the inconvenience of this model can limit its clinical use. We therefore have built a web-based survival risk calculator based on children AML's prediction nomograms. This tool accomplished a successful visualization, and the OS of children with AML was statistically predicted. Finally, an addition to the nomogram was created to differentiate patients at various mortality rates through prognostic risk stratification.

We identified 13 clinicopathological characteristics capable of predicting OS for AML children including gender, age of diagnose, WBC at diagnosis, BM blast percentage, and chromosomal abnormalities [*t*(8; 21), inv(16)]. Several studies have shown that age of diagnose and WBC at diagnosis were important predictive factors [30, 31], while the mechanism remains clear. Further studies are required to identify the mechanisms.

The TARGET database required detailed clinical information such as chemotherapy, which restricted our study of therapeutic modalities' impacts and prognostic complications. Furthermore, due to the retrospective aspect of the analysis, there was a data selection element. The online calculator set up in this thesis can be updated and serves as a foundational resource for further analysis.

## 5. Conclusion

Large data analysis is an important source of clinical prognostic indicators. Some of the latest analyzes of clinical data were focused on the SEER database. The TARGET database is part of the National Cancer Institute project and is barely published on its clinical data. The prognostic nomogram of childhood AML was developed based on the clinical evidence of the patients. Precise assessments of childhood AML will help physicians determine the current state of the individual, choose effective care choices, and establish better follow-up plans.

## Figures and Tables

**Figure 1:** Identification of predictive factors using the Lasso Cox regression. (a) The vertical line was plotted at the given *λ*, selected by cross-validation. For the optimal *λ*, 6 features of them with a nonzero coefficient were selected. (b) The penalization coefficient *λ* in the Lasso model was adjusted using cross-validation and the minimum criterion. The vertical black lines define the optimal *λ*.

**Figure 2:** Predictive nomogram for OS estimation.

**Figure 3:** A dynamic web-based calculator b 95%confidence interval according to the web survival rate calculator.

**Figure 4:** ROC curves and calibration plots of the nomogram in training and validation cohorts. (a) ROC curves for discrimination in the training set. (b) Calibration plot of observed and predicted probabilities for the nomogram in the 3-year training set. (c) Calibration plot of observed and predicted probabilities for the nomogram in the 5-year training set. (d) ROC curves for discrimination in the validation set. (e) Calibration plot of observed and predicted probabilities for the nomogram in the 3-year validation set. (f) Calibration plot of observed and predicted probabilities for the nomogram in the 5-year validation set.

**Figure 5:** (a) Kaplan-Meier survival curves risk score. (b) Kaplan-Meier survival curves of age. (c) Kaplan-Meier survival curves of WBC. (d) Kaplan-Meier survival curves of inv16.

**Table 1:** Clinical characteristics of patients with AML.

Variables	All patients	Training cohort	Validation cohort
	(*N* = 440)	(*n* = 309)	(*n* = 131)
Age			
<14	312 (70.9%)	224 (72.5%)	88 (67.2%)
≥14	128 (29.1%)	85 (27.5%)	43 (32.8%)
Gender			
Male	231 (52.5%)	161 (52.1%)	70 (53.4%)
Female	209 (47.5%)	148 (47.9%)	61 (46.6%)
White blood cell			
<100	363 (82.5%)	254 (82.2%)	109 (83.2%)
≥100	77 (17.5%)	55 (17.8%)	22 (16.8%)
BM leukemic blast percentage			
<90%	333 (75.7%)	255 (82.5%)	78 (59.5%)
≥90%	107 (24.3%)	54 (17.5%)	53 (40.5%)
Chromosomal abnormalities			
*t*(8; 21)	79 (17.9%)	58 (18.8%)	21 (16.1%)
Inv(16)	57 (12.9%)	39 (12.6%)	18 (13.7%)

## Data Availability

The data analyzed were acquired from the Therapeutically Applicable Research To Generate Effective Treatments (TARGET) database (https://ocg.cancer.gov/programs/target).
